The article "The effect of drainage tube on bleeding and prognosis after total knee arthroplasty: a prospective cohort study" was retracted in 2015. Reason: compromised peer review.

# The effect of drainage tube on bleeding and prognosis after total knee arthroplasty: a prospective cohort study

**DOI:** 10.1186/1749-799X-9-27

**Published:** 2014-04-23

**Authors:** Xiao-Han Liu, Pei-Liang Fu, Shi-Ying Wang, Ya-Juan Yang, Gen-Di Lu

**Affiliations:** 1 Department of Nursing, Changzheng Hospital, Second Military Medical University, No. 415 Fengyang Road, Shanghai 200003, China; 2 Department of Joint Surgery, Changzheng Hospital, Second Military Medical University, Shanghai 200003, China

**Keywords:** Total knee arthroplasty, Drainage tube, Bleeding, Prognosis

## Abstract

**Background:**

To evaluate the effect of drainage tube on prognosis after total knee arthroplasty (TKA) and explore an effective treatment with favorable prognosis.

**Methods:**

In a prospective study, 18 patients with TKA for the first time were included and randomly divided into three groups, group A (no placement of drainage tube), group B (negative pressure drainage), and group C (4 h clamping drainage). Intraoperative and postoperative blood loss, operation time, and the drainage volume were recorded and analyzed. Arthrocele, ecchymosis, and range of motion (ROM) were examined postoperatively. The degree of pain was scored by Visual Analog Scale (VAS) after 6, 12, and 24 h of operation. The complications were examined and HSS (hospital for special surgery) knee score was taken during the follow-up period.

**Results:**

There was no significant difference in operation time, total blood loss, intraoperative blood loss, and VAS score among three groups. Meanwhile, the hidden blood loss in group B was significantly decreased compared with group A (*P* = 0.0015). The postoperative drainage volume of group B was significantly increased compared with group C (*P* = 0.0002). No drainage increased the rate of arthrocele and ecchymosis. Compared with group A, ROM after 3 days of operation in groups B and C was significantly increased (*P* = 0.0357, *P* = 0.0372, respectively). During follow-up study, no deep infection or deep venous thrombosis was found.

**Conclusion:**

After TKA, early clamping of the drainage tube reduced the bleeding loss without adverse effect on prognosis, which might be useful for clinical application in future.

## Background

Knee arthroplasty is a surgical procedure to replace the weight-bearing surfaces of the knee joint in order to relieve pain and disability, which is commonly performed for osteoarthritis and rheumatoid arthritis [1]. Since its first performance in 1968, improvements of knee replacement surgery in terms of surgical materials and techniques have greatly increased its effectiveness [2]. According to the Agency for Healthcare Research and Quality, more than 600,000 knee replacements are performed each year in the USA [3]. Knee arthroplasty surgery is performed either as a partial or a total knee arthroplasty (TKA). TKA is a major orthopedic surgery with a closed space, in the form of a new knee joint, and could be performed successfully at all ages [4,5].

Generally, TKA consisted of replacement of the diseased or damaged knee joint surfaces with metal and plastic components allowing continued motion of the knee [6]. Majority of the patients who underwent TKA surgery showed a dramatic reduction of knee pain [7]. However, as an orthopedic surgery with large trauma, the bleeding in TKA is large and mostly occurs after operation by using a tourniquet [8]. The postoperative bleeding is usually drained out via wound drainage and various managements have been reported to improve its effectiveness, such as drain clamping [9].

Clinically, the drainage tube is usually implanted in the wound after TKA surgery and then clamped for several hours to deal with postoperative bleeding, which might reduce the rate of hematoma and the tension of tissue which surrounded wound, ease the pain, and accelerate wound healing [10]. However, postoperative bleeding is proposed in the early stage after operation and as a result, temporary clamping of drains postoperatively is suggested [11,12]. Additionally, the different times of clamping to minimize complications have been differently recommended, and the efficacy of drain clamping on blood loss in postoperative management has not been clearly clarified [4,8,9,13,14].

Moreover, drainage could not completely prevent the formation of hematoma and wound drainage might increase postoperative hemoglobin loss, hospital stay, and the rate of blood transfusion which is associated with serious complications, such as viral infections [8,15]. Consequently, patients might have the sufferings and bear economic loss [16]. Besides, the drainage tube and drain wound might be the potential risk factors for infection, such as retrograde infection of the drainage tube [17]. Therefore, many articles compared the blood loss and infection rates between drained group and non-drained group in order to elucidate the effect of the drain on the prognosis of TKA surgery [18]. However, the comparison results between non-drain and drain are contradictory and more studies are still needed to illustrate the problem.

In the present prospective study, the bleeding and prognosis after TKA were compared among patients who underwent three different draining methods, including no placement of drainage tube, negative pressure drainage, and clamping for 4 h of the drainage. The drain was removed after 24 h of operation. The clinical outcome of three managements was recorded and analyzed, including blood loss and drain volume. After operation, arthrocele, ecchymosis, range of motion (ROM), Visual Analog Scale (VAS) score, deep venous thrombosis, and other complications were assessed. The aim of our study was to explore an effective treatment with less bleeding and favorable prognosis.

## Patients and methods

### Clinical information

This study was a prospective randomized study. From July 2013 to September 2013, a total of 18 patients (4 males and 14 females) who underwent TKA for the first time were included in our study with an average age of 67.2 (range, 60 to 78 years). These patients were randomly divided into three groups by concealed envelopes (*n* = 6), including no placement of drainage tube (group A), negative pressure drainage (group B), and 4 h clamping of drainage (group C). The inclusion criteria were the following: patients with knee osteoarthritis who underwent TKA for the first time; no severe knee varus or valgus (> 15°); no joint flexion contractures; no internal medicine complications, such as the hemorrhagic disease; no diabetes; and a stable blood pressure. The exclusion criteria were the following: patients underwent reversion surgery of the knee, disorder of the blood coagulation system, long-term use of anticoagulants or hormones, infection, and malnutrition. There is no significant difference in the body mass index of patients among these three groups (*P* > 0.05). The present study was approved by the ethics committee of Changzheng Hospital and written informed consent was obtained from all the patients.

### Surgical procedure

The posterior cruciate ligament was used to fix the artificial knee joint (PFC Sigma PS, DePuy, Warsaw, IN, USA). All surgeries were performed by a senior doctor. During the operation, routine tourniquet was used and the volume of bleeding loss was recorded. Then, the tourniquet was released and the bleeding was stopped carefully. The operation time was recorded. Closure was done after inserting a drainage device inside the joint (groups B and C). No drainage was implanted in group A. The standard dressing compression bandage was applied over the dressing. After 24 h of operation, the drainage tube was removed and the drainage volume was measured. The continuous passive motion (CPM) device was used on knee joint after 24 h of operation. Nadroparin calcium and sole vein pump were used to prevent deep vein thrombosis.

The blood loss was measured according to the study of Kim et al. [16]. The hematocrit was examined preoperatively and 24 h postoperatively. In detail, the blood loss was determined using the following formulas: (1) theoretical value blood loss = PBv (preoperative blood volume) × (preoperative hematocrit − postoperative hematocrit), in which PBv = K1 × height (m) + K2 × weight (kg) + K3 (male, K1 = 0.3669, K2 = 0.03219, K3 = 0.6041; female, K1 = 0.3561, K2 = 0.03308, K3 = 0.1833); (2) the actual blood loss = the theoretical value of blood loss + the transfusion volume or the actual blood loss = the dominant blood loss + the hidden blood loss; (3) the dominant blood loss = intraoperative blood loss + postoperative visible blood loss. Intraoperative blood loss was measured by weighing the sponges and measuring the suction bottle. If obvious bleeding occurred postoperatively, transfusion was performed for patients with hemoglobin (Hb) less than 90 g/L.

### Postoperative management

The knee perimeter was measured postoperatively on days 2 and 3. The difference of bilateral knee perimeter of > 1 cm was considered as arthrocele. The petechial area of soft tissue that surrounded knee joint with the size of > 10 cm^2^ was considered as ecchymosis. The maximum flexion angle of knee defined as ROM was measured postoperatively on days 2 and 3.

Celecoxib (200 mg) was taken orally two times a day after operation. For unbearable pain postoperatively, pethidine (100 mg) was intramuscularly injected. The degree of pain was scored by VAS at 6, 12, and 24 h after the operation. Patients in these three groups received the analgesic treatment with oral celecoxib (200 mg each, two times daily). The pain score was measured in resting knee.

The clinical symptoms of deep vein thrombosis were monitored and recorded via color Doppler ultrasonography or angiography. The follow-up period was 4 weeks. The complications were examined and hospital for special surgery (HSS) knee score was determined.

### Statistical analysis

Data were given as mean ± SD in the text. Statistical analysis was performed using SPSS 16.0 software. One-way analysis of variance was used to analyze the difference of measurement data. Chi-square test (*x*^2^ test) was used to analyze the enumeration data. Fisher's exact test was used to compare the differences in the number of arthrocele and ecchymosis. The value of *P* < 0.05 was set as statistically significant.

## Results

The detailed information of detection indexes among groups A, B, and C was shown in Table 1. The operation time ranged from 60 to 90 min, of which no statistical significance was found among three groups. No patient received blood transfusion. The total blood loss in groups A, B, and C was 243 ± 51.30 mL, 270.5 ± 66.11 mL, and 252 ± 25.13 mL, respectively, and there was no significant difference of the total blood loss among three groups. Meanwhile, intraoperative blood loss in groups A, B, and C was 105 ± 57.95 mL, 81.67 ± 57.92 mL, and 99.17 ± 48.85 mL, respectively, and no significant difference was found. Besides, the hidden blood loss in groups A, B, and C was 121.50 ± 43.32 mL, 33 ± 25.44 mL, and 71.83 ± 54.66 mL, respectively, and there was a significant difference between groups A and B (*P* = 0.0015). The postoperative drainage volume of group B (159.17 ± 38.49 mL) was significantly increased compared with that of group C (77.5 ± 33.13 mL) (*P* = 0.0002).

**Table 1:** Comparison of detection indexes among groups A, B, and C

	**Group A**	**Group B**	**Group C**
Patients (M/F)	1/5	3/3	0/6
Operation time (min)	66.17 ± 11.62	66.83 ± 16.50	71.67 ± 13.44
Blood loss			
Total blood loss (mL)	243 ± 51.30	270.50 ± 66.11	252 ± 25.13
Intraoperative blood loss	105 ± 57.95	81.67 ± 57.92	99.17 ± 48.85
Hidden blood loss	121.50 ± 43.32	33 ± 25.44**	71.83 ± 54.66
Drainage volume (mL)		159.17 ± 38.49#	77.5 ± 33.13
VAS			
6 h	2	2	2
12 h	1	1.3 ± 0.47	0.83 ± 0.37
24 h	0.17 ± 0.37	0.5 ± 0.76	0
Complications			
Arthrocele (*n*)	4	1**	1**
Ecchymosis (*n*)	2	0	1
ROM (postoperative)			
2 days	27.5° ± 5.59°	32.5° ± 5.59°	32.5° ± 5.59°
3 days	55° ± 7.07°	66.67° ± 9.43°*	63.33° ± 4.71°*
HSS knee score	83 ± 7	82 ± 5	85 ± 5

*P < 0.05 vs. group A; **P < 0.01 vs. group A; #*P* < 0.05 group B vs. group C. Group A, no placement of drainage tube; group B, negative pressure drainage; group C, 4 h clamping of drainage.

Compared with only one case with arthrocele respectively occurring in groups B and C, four cases showed arthrocele in group A (*P* < 0.01), suggesting that no drainage might increase the rate of arthrocele. No ecchymosis was detected in group B, while two cases and one case showed ecchymosis in groups A and group C, respectively, and no statistical significance was found among three groups. After 2 days of operation, there was no significant difference of ROM among groups A, B, and C (27.5° ± 5.59° vs. 32.5° ± 5.59° vs. 32.5° ± 5.59°). After 3 days of operation, compared with group A, ROM of groups B and C was significantly increased (*P* = 0.0357, *P* = 0.0372, respectively). No statistical significance of VAS score was found among three groups after 6, 12, and 24 h of operation.

During the 4-week follow-up study, no deep infection and no deep venous thrombosis was examined. The HSS knee scores of groups A, B, and C were 83 ± 7, 82 ± 5, and 85 ± 5, respectively, without significant difference.

## Discussion

In this prospective study, bleeding and prognosis after TKA were evaluated among patients with no placement of drainage tube, negative pressure drainage, or 4 h clamping of drainage tube. The clinical outcome of these three managements was analyzed in order to explore an effective treatment with favorable prognosis.

In our study, clamping for 4 h of the drainage tube was set as group C. It had been reported that 37% of blood loss were recorded in the first 2 h after operation and 55% in the first 4 h [19]. As a result, 4 h clamping could represent the outcome of clamping drain. However, the researches of clamping ranging from 1 to 24 h showed inconsistent effectiveness and patients with wide range of age and in the degree of knee dysfunction are still needed to enroll.

Compared with group A, no significant difference of total blood loss and intraoperative blood loss was found among the three groups. Besides, there was significant difference of hidden blood loss between groups A and B (*P* = 0.0015). These results suggested that blood loss of drainage group (group B and C) was slightly higher than that of non-drainage group (group A). Our results coincided with the previous studies. Tai et al. [15] have suggested that postoperative hemoglobin loss of drain clamping group (clamping in the first 4 h post operation) was more than that of non-drain group. However, Mengal et al. [18] have reported that the wound drainage did not lead to increase blood loss and non-drainage did not reduce blood loss. These contradictions might be associated with the clinical features of the patients. Besides, it has been suggested that the hidden loss might be nearly 50% of the total loss [20], which should be taken into account when managing blood loss after TKA [21]. The hidden blood loss in TKA might be promoted by using a tourniquet [22]. The postoperative drainage volume of group B (negative pressure drainage) was significantly increased compared with that of group C (clamping for 4 h) (*P* = 0.0002) in our study. The increased blood loss in group B might be due to the pressure drop and the disappeared tamponade of hematoma inside the wound [23]. The decreased blood loss in group C might be associated with the temporary tamponade of hematoma inside the wound [15]. Unfortunately, the symptoms, such as swelling and hematoma, were very difficult to standardize as indicators for hidden blood loss [24].

For the postoperative curative effect, arthrocele (four cases) and ecchymosis (two cases) were detected in non-drainage group, while ROM after 3 days of operation was significantly increased in the drainage group, compared with the non-drainage group. All these outcomes might be due to the tamponade of hematoma in the wound. Previous studies theorized that postoperative bleeding might be decreased by the tamponade effect that occurred when a drain was eliminated and a compressive dressing was applied [13]. Besides, the drain might prevent the formation of a hematoma which could inhibit wound healing and increase the deep infection rate [23]. Other factors of blood loss include gender [25], obesity [20], and use of tranexamic acid [26].

During the follow-up study, no deep infection and no deep venous thrombosis were found among the three groups. Besides, no significant difference of HSS knee score was identified. Our results demonstrated the safety and effectiveness of drainage and non-drainage to some extent. However, long-term follow-up was still needed to monitor the prognosis of TKA. Huang et al. [27] have retrospectively reviewed 25 cases of high-flex TKA with a minimum follow-up of 2 years. Besides, Callaghan et al. [28] have reported a 9- to 12-year follow-up of patients who had a primary total knee replacement performed with cemented rotating platform. Moreover, the enrolled patients were further divided into three groups leading to smaller numbers. Therefore, a larger sample size is needed to further evaluate the effect of drainage tube on the prognosis after TKA and explore an effective treatment with favorable prognosis.

## Conclusions

The blood loss was reduced in non-drainage group, accompanied by postoperative discomfort in early stage. Compared with negative pressure drainage, clamping for 4 h of the drainage tube showed reduced blood loss without significant difference of the prognosis, suggesting that early clamping of drainage tube was a benefit to the reduction of blood loss and did not adversely influence the recovery of joint function. Our study provided the basis for exploring an effective procedure of TKA.

## Abbreviations

CPM: continuous passive motion; Hb: hemoglobin; HSS: Hospital for Special Surgery; ROM: range of motion; TKA: total knee arthroplasty; VAS: Visual Analog Scale.

## Competing interests

The authors declare that they have no competing interests.

## Authors’ contributions

GDL and XHL conceived and designed the experiments. XHL, PLF, SYW, and YJY acquired and analyzed the data: GDL drafted and approved the manuscript. All authors read and approved the final manuscript.
